The article "Effects of Naturally Occurring Six- and Twelve-Nucleotide Inserts on Newcastle Disease Virus Replication and Pathogenesis" was retracted in 2020. Reasons: manipulated images; duplicated images; concerns about the data.

# Effects of Naturally Occurring Six- and Twelve-Nucleotide Inserts on Newcastle Disease Virus Replication and Pathogenesis

**DOI:** 10.1371/journal.pone.0103951

**Published:** 2014-08-05

**Authors:** Anandan Paldurai, Sa Xiao, Shin-Hee Kim, Sachin Kumar, Baibaswata Nayak, Sweety Samal, Peter L. Collins, Siba K. Samal

**Affiliations:** 1 Virginia-Maryland Regional College of Veterinary Medicine, University of Maryland, College Park, Maryland, United States of America; 2 Laboratory of Infectious Diseases, National Institute of Allergy and Infectious Diseases, Bethesda, Maryland, United States of America; University of Rochester Medical Center, United States of America

## Abstract

Newcastle disease virus (NDV) isolates contain genomes of 15,186, 15,192 or 15,198 nucleotides (nt). The length differences reflect a 6-nt insert in the 5′ (downstream) non-translated region (NTR) of the N gene (15,192-nt genome) or a 12-nt insert in the ORF encoding the P and V proteins (causing a 4-amino acid insert; 15,198-nt genome). We evaluated the role of these inserts in the N and P genes on viral replication and pathogenicity by inserting them into genomes of two NDV strains that have natural genome lengths of 15,186 nt and represent two different pathotypes, namely the mesogenic strain Beaudette C (BC) and the velogenic strain GB Texas (GBT). Our results showed that the 6-nt and 12-nt inserts did not detectably affect N gene expression or P protein function. The inserts had no effect on the replication or virulence of the highly virulent GBT strain but showed modest degree of attenuation in mesogenic strain BC. We also deleted a naturally-occurring 6-nt insertion in the N gene from a highly virulent 15,192-nt genome-length virus, strain Banjarmasin. This resulted in reduced replication *in vitro* and reduced virulence *in vivo*. Thus, although these inserts had no evident effect on gene expression, protein function, or replication *in vivo*, they did affect virulence in two of the three tested strains.

## Introduction

Newcastle disease (ND) is one of the most important diseases of domesticated and wild birds [1], [2]. The causative agent ND virus (NDV) causes a highly contagious and lethal disease that accounts for huge economic losses to the poultry industry worldwide [1]–[3]. NDV is a single stranded negative sense RNA virus in the genus *Avulavirus* under the family *Paramyxoviridae* [4], [5]. The genome of NDV contains six genes encoding the nucleocapsid protein (N), phosphoprotein (P), matrix protein (M), fusion protein (F), hemagglutinin-neuraminidase protein (HN), and large polymerase protein (L). In addition, the P gene encodes an additional protein called V that is expressed by RNA editing.

The article "Effects of Naturally Occurring Six- and Twelve-Nucleotide Inserts on Newcastle Disease Virus Replication and Pathogenesis" was retracted in 2020. Reasons: manipulated images; duplicated images; concerns about the data.

Naturally occurring NDV strains exhibit a spectrum of virulence, with mortality in chickens ranging from 0 to 100% [1]–[3]. Based on the degree of virulence, NDV strains are classified as lentogenic (low virulence), mesogenic (moderate virulence) and velogenic (high virulence) pathotypes [1]–[3]. In addition, NDV strains are categorized into two phylogenetically divergent classes, namely class I and class II. Class I strains are typically isolated from healthy water fowl and are not associated with disease. Class II contains strains that cause infections ranging from inapparent to highly fatal. These two classes are further divided into genotypes based on partial or complete nucleotide sequence of the F gene. Currently, class I strains represent a single genotype and class II strains represent at least XVIII genotypes [6]–[9].

The complete genome sequence analysis of NDV strains reveal the existence of genome lengths of 15,186 nucleotides (nt) [2], [4], [10]–[12], 15,192 nt [13]–[15] or 15,198 nt [16]–[20]. All these genome lengths are divisible by six conforming to the ‘rule of six’ that is observed in all viruses of the subfamily *Paramyxovirinae* [4]. These sequence length variations in the NDV genome was identified in the nucleoprotein gene and in the phosphoprotein gene as a 6-nt and 12-nt insert sequences, respectively. Previous studies involving genome sequence analysis of NDV strains identified the presence of the N-gene and P-gene inserts and related them to the natural history of NDV as: the 15,186-nt genome-length viruses circulated between 1930 and 1960, and the 15,192-nt and 15,198-nt genome-length viruses emerged after 1960 [10]–[20]. The 15,186-nt and 15,192-nt genome-length viruses belong to the NDV genetic class II and the 15,198-nt genome-length viruses belong to NDV genetic class I. Currently, all three genome-length viruses are circulating in bird populations around the world. The sequence alignment and phylogenetic tree analysis revealed that NDV strains which belonged to a particular genome-length assignment clustered together (Fig. 1). The percent nt sequence identities of NDV genomes suggest a very close genetic relationship of a particular genome-length virus strains to others (Table S1). In addition, our laboratory recently identified a unique virus of the 15,198-nt genome-length containing a 6-nt insert in the N gene and another 6-nt insert in the intergenic sequence between HN and L genes [22]. This later HN-L insert will not be addressed in the present study.

**Figure 1:** Nucleotide sequence alignment and phylogenetic tree analysis of NDV strains. (a) Nucleotide (nt) sequence alignment of part of the 5′ (downstream) non-translated region (NTR) of the Nucleocapsid protein (N) gene of NDV strains to illustrate the 6-nt insert that is characteristic of 15,192-nt size class viruses. (b) Nt sequence alignment of part of the ORF of the Phosphoprotein (P) gene NDV strains to illustrate the 12-nt insert that is found in many of the 15,198-nt size class viruses. All sequences shown are negative-sense and gaps indicate absence of the insert sequence. The nucleotide residues are color coded; U-violet, A-green, G-yellow and C-blue. (c) Phylogenetic tree analysis based on the nt sequences of complete genomes of NDV strains. Note the clustering of NDV strains with respect to their genome-length. Branches in each cluster is color coded: red-15,186 nt; green-15,192 nt; blue-15,198 nt. The tree was constructed by bootstrap analysis (1000 replications) using the neighbor-joining of the Kimura-2-parameter method for nt differences in the MEGA 4.0 phylogenetic analysis program [21]. Scale bar shows number of base substitutions per site. Bootstrap values are shown at the nodes. Note the clustering of unique genome-length viruses. Asterisk (*) indicate the reference for the sequence of strain BC [11]. The genetic class designations are indicated for NDV strains in all three panels.

The article "Effects of Naturally Occurring Six- and Twelve-Nucleotide Inserts on Newcastle Disease Virus Replication and Pathogenesis" was retracted in 2020. Reasons: manipulated images; duplicated images; concerns about the data.

All the 15,192-nt genome-length viruses contain a 6-nt insert (e.g., AGGGUG in strain ZJ1) in the 5′ (downstream) noncoding region of the N gene after genome position 1647 [13], [14] (Fig. 1a), and all previously-analyzed 15,198-nt genome-length viruses contain a 12-nt insert (e.g., ACCCUCUGCCCC in strain Alaska 415) in the ORF encoding the P and V proteins after genome position 2381 [16]–[20]. The 12-nt insertion increases the lengths of the P and V proteins by four amino acids (aa) without affecting their reading frames. The aa sequence introduced in P and V proteins are WETG and VGDG, respectively, at aa position 166 to 169 (e.g., strain Alaska 415). The importance of these inserts in NDV biology is not known.

In this study, we investigated the biological significance of the 6-nt N and 12-nt P inserts by introducing them separately by reverse genetics into the genomes of two genetically cloned 15,186-nt genome-length viruses strain Beaudette C (BC) [11], [23] and strain Texas GB (GBT) [24]. Reciprocally, we also evaluated the effect of deleting the 6-nt N insert from a naturally-occurring 15,192-nt genome-length strain Banjarmasin (Ban) [25], [26]. The strains BC and GBT are genetically closely related and belong to genotype II, and the strain Ban belongs to genotype VII. All three strains belong to NDV phylogenetic class II and possess an identical sequence ^112^RRQKR↓F^117^ at the proteolytic cleavage site of their fusion proteins but differ in virulence. BC is a mesogenic strain and GBT and Ban are velogenic strains.

The article "Effects of Naturally Occurring Six- and Twelve-Nucleotide Inserts on Newcastle Disease Virus Replication and Pathogenesis" was retracted in 2020. Reasons: manipulated images; duplicated images; concerns about the data.

Our results showed that the addition of the 6-nt N or the 12-nt P insert into the genome of 15,186-nt genome-length viruses or the deletion of the 6-nt insert from a 15,192-nt genome virus resulted in a decrease of virulence. These results suggest that the 6-nt and the 12-nt inserts found in the 15,192-nt and 15,198-nt genome-length viruses may not have any direct role in replication and virulence but they make up the optimal genome-length that is required for efficient virus replication and pathogenesis.

## Materials and Methods

### Cells and viruses

A chicken embryo fibroblast cell line (DF-1), a human epidermoid carcinoma cell line (HEp-2), and a human embryonic kidney cell line (293T) were obtained from the American Type Culture Collection (ATCC, Manassas, VA). The cell lines were grown in Dulbecco’s minimal essential medium (DMEM) with 10% fetal bovine serum (FBS) and maintained in DMEM with 2% FBS. The modified vaccinia virus strain Ankara (MVA) expressing T7 RNA polymerase was kindly provided by Dr. Bernard Moss (NIH, Bethesda, MD). The recombinant (r) NDV strains BC (rBC), GBT (rGBT), Banjarmasin (rBan), and their mutant derivatives were grown in nine-day-old embryonated specific-pathogen-free (SPF) chicken eggs in an enhanced biosafety level 3 (BSL-3+) containment facility certified by the USDA following the guidelines of the IACUC, University of Maryland.

### Reverse genetic systems for NDV strains BC, GBT, and Ban

Full-length antigenome cDNA clones of NDV strains BC and GBT were constructed in the present study by sequential cloning into pBR322/HDr vector using a previously-described strategy [23]. First a 112 nt linker sequence containing 9 unique restriction enzyme (RE) sites in the order of AscI, PacI, PmeI, AsiSI, AgeI, SnaBI, BstBI, MluI and RsrII, was cloned between AscI and RsrII sites in the pBR322/HDr vector. Among these RE sites, AgeI site was a unique site present in the genomes of BC and GBT. The antigenomes of BC and GBT were constructed as 8 matching fragments using the 9 restriction enzyme sites noted above, which were spaced identically in each antigenome construct (Fig. 2a). The segments were synthesized by PCR from BC full length plasmid DNA [23] and from viral RNA using RT-PCR for GBT. PCR was performed with the high fidelity platinum *Pfx* polymerase, and the gel purified fragments were digested and sequentially cloned into the pBR322/HDr vector [23]. The sequential cloning of N, P, M, F and HN genes was performed as segments 1, 2, 3, 4 and 5. The L gene was cloned as three fragments, namely, 6, 7 and 8. In total, 16 nt changes were introduced in the antigenomes of strains BC and GBT to introduce the RE sites and to modify a naturally occurring RsrII site in the P gene. All of the RE sites were introduced into non-translated regions with the exception of the BstBI and MluI sites that were introduced into the L ORF. The nt changes in the L ORF were introduced in such a way that the aa sequence was not altered. The nt changes made are A(1768)T, C(1769)T, C(1773)T, A(3221)G, A(3222)T, T(3227)A, T(4452)G, T(4453)C, T(4457)C, A(4458)G, T(4459)C, A(8327)C, G(8330)A, G(10396)A, A(13537)G, and A(13537)G. Support plasmids expressing the N, P, and L proteins of strain GBT were constructed using the pGEM7Z (+) expression vector. Support plasmids for NDV strains BC and Ban were previously constructed in our laboratory [23], [25].

The article "Effects of Naturally Occurring Six- and Twelve-Nucleotide Inserts on Newcastle Disease Virus Replication and Pathogenesis" was retracted in 2020. Reasons: manipulated images; duplicated images; concerns about the data.

**Figure 2:** Gene map, reverse genetic cloning strategy for NDV strains Beaudette C, GB Texas and Banjarmasin. (a) Gene map and cloning strategy for NDV strains BC and GBT and their mutant viruses. Top two schematic gene maps show genetic structure, genome-length and cloning strategy for NDV strains BC and GBT. The location of RE sites in the antigenome cDNA clones of strains BC and GBT are shown. The numerals indicate genome nt position. AscI and RsrII sites are present before T7 promoter (T7pr) sequence and within hepatitis delta virus ribozyme/T7 terminator (HDr/T7tr) sequence, respectively, in the plasmid vector pBR322 (see Materials and Methods section). Bottom six gene maps illustrate the recombinant, 6-nt and 12-nt insert mutant viruses. The diagrams of N and P gene boxes show the position (indicated by a small box in black) of the 6-nt and 12-nt inserts in rBC and rGBT to generate mutant viruses rGBT-N6 and rBC-N6 (genome lengths of 15,192 nt) and rGBT-P12 and rBC-P12 (genome lengths of 15,198 nt). The nt position and sequence of the insert is given on the left. (b) Gene map of recombinant and 6-nt deletion mutant of NDV strain Ban. The recombinant and the 6-nt deleted viruses are indicated by rBan and rBan-ΔN6, respectively. The deleted 6-nt sequence and the nt position (indicated by a small box in black) in the 15,192-nt genome of Ban is provided on the left. Le and Tr indicate leader and trailer regions, respectively.

### Construction and rescue of mutant viruses of NDV strains BC, GBT, and Ban

A 6-nt (AGGGUG) or 12-nt (ACCCUCUGCCCC) insert conforming to the respective consensus sequence (see Results and Fig. 2a) was introduced separately into the N (after nt position 1647) or P (after nt position 2381) genes of strains BC and GBT using overlap PCR and cloned using RE sites AscI and PacI for N gene and PacI and PmeI for P gene, respectively. In addition, the existing 6-nt N insert that occurs naturally in strain Ban was deleted by the same method using RE sites AscI and PacI (Fig. 2b).

The article "Effects of Naturally Occurring Six- and Twelve-Nucleotide Inserts on Newcastle Disease Virus Replication and Pathogenesis" was retracted in 2020. Reasons: manipulated images; duplicated images; concerns about the data.

### Virus growth kinetics and plaque morphology

The growth kinetics of rBC, rGBT, rBan, and their mutant viruses were determined under multi-cycle growth conditions in DF-1 cells. The virus was inoculated at a multiplicity of infection (MOI) of 0.01 PFU into DF-1 cells grown in DMEM with 10% FBS at 37°C. Aliquots from the medium supernatant were collected at 8-h intervals until 64 h post infection for rBC and rGBT viruses and their mutants (Fig. 3a, b). For rBan and its mutant, DF-1 cells were infected with an MOI of 0.01 PFU, and aliquots from the medium supernatant were collected at 12 h intervals for 48 h (Fig. 3c). Viral titers were assayed by limiting dilution in DF-1 cells, and titers were determined using the method of Reed and Muench [27] and expressed as 50%-tissue-culture-infectious-dose (TCID50) units. Plaque assays were performed to determine the plaque morphology: plaques were photographed and measured on day 5 in the case of the rBC and rGBT groups of viruses, and on day 7 for rBan and its mutant virus (Fig. 3d).

**Figure 3:** Growth kinetics and plaque morphology of recombinant NDV strains in chicken embryo fibroblast (DF-1) cells. The multi-cycle growth kinetics of recombinant BC (rBC) (a), GBT (rGBT) (b) and Ban (rBan) (c) in parallel with their mutant viruses in DF-1 cells. Values are the means of triplicate wells. Error bars indicate mean±SEM. (d) Plaque morphology of rBC, rGBT and rBan group viruses in DF-1 cells. Note the larger plaque size of GBT and Ban viruses compared to BC viruses, and the similarity between the mutant viruses and their parents.

### Production of N protein antiserum and immunoblot analysis

A 15-aa synthetic peptide was custom synthesized (GenScript) in which first aa was an added cysteine for conjugation and aa 2 to 15 corresponded to aa 191 to 204 of the N protein of NDV strain LaSota. One rabbit was injected with 1 mg of KLH-conjugated synthetic N protein peptide in Freund's complete adjuvant to raise anti-N protein antiserum. After 2 weeks, a booster immunization was given with 0.5 mg of the peptide in Freund's incomplete adjuvant, and the hyperimmune serum was collected 2 weeks later. Western blot analysis was performed using NDV-infected cell lysates to confirm the specificity of the antisera to NDV N protein (data not shown).

Expression of N protein in the recombinant viruses, rBC and rBC-N6 and rBan and rBan-ΔN6, were examined by immunoblot analysis. Briefly, DF-1 cells were infected at a MOI of 0.1 PFU. The cells were harvested at 24 h post infection, the lysed proteins were denatured, reduced, separated by NuPAGE 4–12% Bis-Tris gel (Life Technologies, Grand Island, New York), and analyzed by immunoblotting using a 1∶100 dilution of anti-N peptide antibody described above. β-Tubulin was used as the loading control. The band density of N protein was quantitated and compared between rBC and rBC-N6 and between rBan and rBan-ΔN6 using ImageJ analysis [28] (Fig. 4a, b).

The article "Effects of Naturally Occurring Six- and Twelve-Nucleotide Inserts on Newcastle Disease Virus Replication and Pathogenesis" was retracted in 2020. Reasons: manipulated images; duplicated images; concerns about the data.

**Figure 4:** Comparative analysis of nucleocapsid protein expression and phosphoprotein function. (a) Nucleocapsid protein expression in DF-1 cells infected with rBC and rBC-N6 and rBan and rBan-ΔN6. Replicate cell monolayers were infected with rBC and rBC-N6 and rBan and rBan-ΔN6 at an MOI of 0.1, and were harvested at 24 h post-infection. Cell lysates were prepared and analyzed by polyacrylamide gel electrophoresis and immunoblotting with a polyclonal serum against a peptide prepared from the sequence of the N protein. β-Tubulin was used as the loading control. (b) The density of the N protein bands at 24 h was quantified to compare the N protein expression between parental viruses rBC and rBan to their respective N6 and ΔN6 mutant viruses using ImageJ program [28]. Note the similarity between the band densities of rBC and BC-N6 and rBan and rBan-ΔN6. (c) Map of the cDNA encoding the BC minigenome, which consisted of the first 166 nt from the leader end of the BC genome, followed by the CAT ORF, followed by the last 152 nt of the trailer end of the BC genome. (d) Analysis of mini-genome activity in lysates from transfected cells using an ELISA for the CAT protein to compare the activities of the wt and P12 versions of the P protein of strain BC. The N+P and N+P12 transfections are negative controls. CAT expression was expressed as absorbance at 405 nm.

### Minigenome system for NDV strain BC

We developed a minigenome system for strain BC. A cDNA was designed to encode a negative-sense mini-genome containing (Fig. 4c): the 3′-terminal 221 nt of the BC genome, including the 55-nt leader region and complete upstream non-translated region of N gene, followed by the 660-nt chloramphenicol acetyl transferase (CAT) reporter gene in negative sense, followed by the 5′-terminal 265 nt of the BC genome, including the last 152 nt of the L gene (containing the last 42 nt of the coding region and the complete downstream non translated region) and the 113-nt trailer region. In the mini-genome cDNA, the leader region was flanked by the hepatitis delta virus ribozyme and the trailer was flanked by a T7 promoter sequence, so that T7 transcription would yield a negative-sense mini-genome (Fig. 4c). The minigenome cDNA was constructed from three fragments containing (i) the leader and upstream N sequence, (ii) the CAT sequence, and (iii) the downstream L and trailer sequence. These three fragments were joined sequentially by two rounds of overlapping PCR using high fidelity *Pfx* polymerase. The final product was cloned into pBR322/HDr between RE sites AscI and RsrII as shown in Figure 4c, and its sequence was confirmed.

The article "Effects of Naturally Occurring Six- and Twelve-Nucleotide Inserts on Newcastle Disease Virus Replication and Pathogenesis" was retracted in 2020. Reasons: manipulated images; duplicated images; concerns about the data.

Expression plasmids of BC N, P, L, and P with 12 nt insertion also were cloned separately in pCDNA3.1 (+) expression vector. 0.8 µg of minigenome plasmid and 0.8 µg of N, 0.6 µg of P or P with 12 nt insert (P12) and 0.5 µg of L plasmids were transfected using Lipofectamine 2000 reagent on to a 80% monolayer of 293T cells in 12-well cell culture plate. MVA-T7 was used to infect the monolayer at the same time. Media was changed after 3 h, and incubated for 48 h and samples for CAT-ELISA were processed following the manufacturer’s protocol and the OD values were recorded at 405 nm (Fig. 4d). Plasmids N and P were used along with BC minigenome to serve as control.

### Pathogenicity studies

The pathogenicity of the parental and mutant viruses was quantified by the MDT test in nine-day-old embryonated chicken eggs and the ICPI test in one-day-old chicks [3]. To evaluate replication and pathogenicity of the rBC and rGBT viruses and their mutant derivatives in birds, two-week-old SPF chickens in groups of 13 were inoculated with 0.2 ml of 10^6^ PFU of each virus by the oculonasal route. Three birds from each group were euthanized at 3 DPI and tissues from lung, trachea, spleen, brain and intestine were collected. For virus titration, the tissue samples were homogenized, and the supernatant was serially diluted and used to infect DF-1 cells, with duplicate wells per dilution. Infected wells were identified by HA assay of the supernatant, and the titer was calculated using the method of Reed and Muench [27] and expressed as TCID50/g of tissue (Fig. 5).

**Figure 5:** Virus titers of rBC and rGBT and their mutants in two-week-old chickens following oculonasal inoculation. Tissue samples from the trachea, lungs, spleen, intestine, and brain of 3 chickens (n = 3) from each indicated virus group were harvested on day 3 post infection, and virus titers were determined by limiting dilution assay [27]. The mean virus titer from 3 chickens per group was given for each tissue sample. Error bars indicate mean±SEM.

The remaining 10 chickens in each group were observed for clinical signs of disease until 14 days post infection (DPI). The birds were scored daily as follows: 0 for normal, 1 for sick, 2 for paralysis/twitching/wing drop, 3 for prostration, and 4 for death. A mean score per virus group per day was generated for comparison. The mortality pattern was observed daily for the entire 14 days to generate the survival pattern of chickens among the virus groups (See Results and Fig. 6).

The article "Effects of Naturally Occurring Six- and Twelve-Nucleotide Inserts on Newcastle Disease Virus Replication and Pathogenesis" was retracted in 2020. Reasons: manipulated images; duplicated images; concerns about the data.

**Figure 6:** Percent survival and clinical score curves for recombinant and mutant viruses. Percent survival curve and clinical score curves for recombinant NDV strains BC (a, b), GBT (c, d) and Ban (e, f) in two-week-old chickens following oculonasal inoculation. The birds (10 per group) were clinically scored for 14 days using a scoring system for the clinical signs: 0, normal; 1, sick; 2, paralysis/twitching/wing drop; 3, prostration; and 4, death. The mean scores per group per day are plotted in the graph.

For rBan and its mutant virus, chickens in groups of 10 were inoculated with 0.2 ml of 2×10^4^ PFU of virus by the oculonasal route. This lower dose (compared to the BC and GBT groups) was used because of the greater virulence of rBan. The birds in each group were observed daily for 14 days and scored for disease as described for the rBC and rGBT groups (Fig. 6).

For *in vivo* experiments, nine-day-old embryonated chicken eggs (MDT assay), one-day-old White Leghorn chicks (ICPI assay), and two-week-old White Leghorn chickens (Pathogenesis study) were used. A New Zealand White rabbit was used for the immunization study. The chicken eggs and the animals were SPF and were procured from the Sunrise Farms Inc., Stuarts Draft, Virginia and from the Charles River Laboratories, Germantown, Maryland, respectively. The animals were housed and cared for in accordance with established guidelines, and the experimental procedures were performed with approval from Institutional Animal Care and Use Committee of the University of Maryland. The end point for all the *in vivo* experiments was death but chicks in ICPI assay and chickens in the pathogenesis study that showed terminal signs of disease. For example, chickens showing paralysis and movement restriction, were euthanized using a higher dose of gaseous anesthetic Isoflurane.

### Ethics Statement

All pathogenicity studies were conducted under biosafety level (BSL3)-enhanced conditions at the University of Maryland. Animals were cared for in accordance with established guidelines, and the experimental procedures were performed with approval from Institutional Animal Care and Use Committee of the University of Maryland, protocol number R-12–93.

### Statistical analysis

Statistically significant differences in data from different recombinant virus groups were evaluated by one-way analysis of variance (ANOVA). Growth kinetics for various groups were analyzed using correlation of XY pairs (Pearson) and P value (two tailed). P values below 0.05 were regarded as being significant for all analyses. Experiments were repeated a minimum of three times. Statistical analysis for mean and standard deviation of data and one-way ANOVA was done by using Prism 5.0 computer software (GraphPad Software Inc., San Diego, CA).

The article "Effects of Naturally Occurring Six- and Twelve-Nucleotide Inserts on Newcastle Disease Virus Replication and Pathogenesis" was retracted in 2020. Reasons: manipulated images; duplicated images; concerns about the data.

## Results

### Design and rescue of recombinant wild type and mutant viruses

In the present study, we investigated the functional significance of the 6-nt insert in the N gene and the 12-nt insert in the P gene by introducing them separately by reverse genetics into the genomes of two 15,186-nt genome-length viruses representing two different NDV pathotypes, namely the moderately virulent strain BC and the highly virulent strain GBT. Consensus sequences for the 6- and 12-nt inserts were determined by aligning the sequences of the N and P genes of representative 15,192- and 15,198-nt genome-length NDV strains (Fig. 1a, b). This showed that the 6-nt insert had conserved residues at positions 2, 3 and 4 (−GGG−) (Fig. 1; sequences are negative sense), while the 12-nt insert was found conserved in the representative strains (ACCCUCUGCCCC) (Fig. 1b). We therefore chose the 6-nt sequence AGGGUG and the 12-nt sequence ACCCUCUGCCCC for insertion into BC and GBT. We also performed deletion of a naturally occurring 6-nt insert (GGGGCG) from the N gene 5′NTR of a velogenic NDV strain Ban containing 15,192-nt genome-length [25].

We constructed and recovered the wild type (wt) viruses rBC and rGBT, which are recombinant versions of strains BC and GBT (Fig. 2a). We then constructed and recovered the mutant derivatives rBC-N6 and rGBT-N6, in which the 6-nt insert AGGGUG was inserted into the N gene after position 1647 (resulting in viral genomes of 15,192 nt) (Fig. 2a). We also constructed the mutant derivatives rBC-P12 and rGBT-P12, in which the 12-nt insert ACCCUCUGCCC was inserted into the P gene after position 2381 (resulting in viral genomes of 15,198 nt) (Fig. 2a). The parental recombinant and genome-length mutant viruses were serially passaged 5 times in nine-day-old embryonated chicken eggs and 5 times in chicken embryo fibroblast DF-1 cells and the stability of the created restriction enzyme sites and insert sequences were confirmed by sequence analysis.

We previously developed a reverse genetic system for the virulent 15,192-nt genome-length strain Ban [25], which has a naturally-occurring 6-nt insert (GGGGCG from genome nt position 1648–1653) in the N gene. We used this system to delete the 6-nt sequence resulting in the virus rBan-ΔN6 (to generate a 15,186 nt genome) (Fig. 2b). This virus also was passaged 5 times in embryonated eggs and its sequence confirmed.

The article "Effects of Naturally Occurring Six- and Twelve-Nucleotide Inserts on Newcastle Disease Virus Replication and Pathogenesis" was retracted in 2020. Reasons: manipulated images; duplicated images; concerns about the data.

### Multi-cycle growth kinetics and plaque morphology

The multi-cycle growth kinetics and plaque morphology of the N6 and P12 mutant viruses were evaluated *in vitro* in DF-1 cells using standard procedures [23]. The growth kinetics and titers of BC N6 and P12 derivatives were relatively similar compared to their parental biological and recombinant BC parents and reached their maximum titers at 32 h post infection (PI) (Fig. 3a). The biological and recombinant versions of the parental GBT strain (wt GBT and rGBT, respectively) had similar growth patterns and plaque morphologies (data not shown). Compared with the parental viruses, rGBT-N6 and rGBT-P12 had very similar growth kinetics throughout the course of 64 h PI and reached maximum titers at 24 h indicating a higher growth kinetics than BC viruses (Fig. 3b). The rBan and rBan-ΔN6 viruses had similar growth kinetics at 12 and 24 h, but at later times, i.e., in 36 and 48 h the mean titer (log_10_ TCID50/mL) of rBan was 7.25 and 8.2 compared to 6.9 and 7.6 of rBan-ΔN6, respectively (Fig. 3c). The plaque sizes of the various viruses were compared by measuring the diameters of 20 randomly picked plaques for each virus. The mean plaque diameters (in mm) were: 1.83±0.12, 1.76±0.1 and 1.87±0.15 for rBC, rBC-N6 and rBC-P12, respectively; and 2.82±0.16, 2.91±0.19 and 2.87±0.17 for rGBT, rGBT-N6, and rGBT-P12, respectively (Fig. 3d). Thus, there were no significant differences in plaque size between the mutant viruses and their respective parental recombinant viruses, although overall the plaque sizes of the BC viruses were substantially less than those of the GBT viruses. The plaques produced by the rBan and rBan-ΔN6 viruses were large and relatively similar in size with a diameter of 2.95±0.31 and 3.12±0.23 mm, respectively (Fig. 3d).

### Immunoblot analysis for nucleocapsid protein expression

To investigate the influence of the 6-nt insert in the N gene (which occurred in the downstream non-translated sequence) on N protein expression, replicate DF-1 monolayers were infected with 0.1 MOI of the rBC and rBC-N6 and rBan and rBan-ΔN6 viruses, and cells were harvested at 24 h, and lysates were prepared and analyzed by gel electrophoresis (Fig. 4a). The relative band densities for rBC and rBC-N6 and rBan and rBan-ΔN6 were 1.0 and 0.987 and 1.0 and 1.064, respectively, suggesting no apparent difference in expression levels between the rBC and rBC-N6 viruses and between the rBan and rBan-ΔN6 viruses (Fig. 4b).

### BC mini-genome CAT reporter gene assay for P protein function

To evaluate the effect of the 12-nt insertion in the P gene (which occurred within the ORF and added 4 aa to P and V), we developed a mini-genome system for strain BC. In this system, a mini-genome cDNA was constructed to encode a negative-sense genome analog that contained the 3′ leader and 5′ trailer regions of strain BC flanking a negative-sense copy of the CAT gene under the control of BC gene-start and gene-end transcription signals (Fig. 4c). This was transfected into 293T cells together with N, P, and L support plasmids (namely, pN, pP and pL) and MVA-T7 vaccinia virus, and at 48 h the cells were harvested and assayed for CAT expression by ELISA. The minigenome complemented with wt pN, pP and pL yielded a mean OD value of 2.412 and with pN, pP12 (12-nt in P gene ORF) and pL resulted in a mean OD value of 2.462 (Fig. 4d). Negative controls in which the BC minigenome was complemented with pN and pP or with pN and pP12 yielded mean OD values of 0.186 and 0.158, respectively. The close similarity between the transfections with wt P compared to mutant P12 indicated that the insertion of 4 aa within the P protein did not affect its function.

The article "Effects of Naturally Occurring Six- and Twelve-Nucleotide Inserts on Newcastle Disease Virus Replication and Pathogenesis" was retracted in 2020. Reasons: manipulated images; duplicated images; concerns about the data.

### Mean death time (MDT) and intracerebral pathogenicity index (ICPI)

To determine the effect of the 6-nt and 12-nt inserts on the virulence of NDV, the parental and mutant viruses were evaluated for MDT in nine-day-old embryonated chicken eggs and for ICPI in one-day-old chicks (Table 1). The MDT and ICPI values of the biological wt versus the recombinant wt viruses of strains BC and GBT were similar, indicating that the recombinant viruses retained the pathogenicity phenotype of the biological parents. The mutant viruses (rBC-N6, rBC-P12, rGBT-N6, and GBT-P12) also had MDT values similar to those of their respective parental biological and recombinant viruses (Table 1). In contrast, the MDT value of the ΔN6 virus was higher than that of rBan, indicative of a decrease in virulence (Table 1).

**Table 1:** Mean death time (MDT) assay and intracerebral pathogenicity index (ICPI) assay scores of parental and N6 and P12 mutant viruses of NDV strains Beaudette C (BC), Texas GB (GBT) and Banjarmasin (Ban).

Virus	MDT (h)*	ICPI score#
wtBC	60±2.0	1.60±0.020
rBC	59±1.0	1.58±0.035
rBC-N6	58±1.5	1.54±0.010
rBC-P12	61±3.0	1.52±0.045
wtGBT	48±1.0	1.90±0.020
rGBT	47±1.5	1.88±0.035
rGBT-N6	46±0.5	1.90±0.015
rGBT-P12	47±1.0	1.86±0.020
rBan	52±2.0	1.81±0.025
rBan-ΔN6	56±1.0	1.68±0.135

*Pathotype definitions by MDT: >90 h, lentogenic; 60 to 90 h, mesogenic; <60 h, velogenic.

# Pathotype definitions by ICPI: velogenic strains approach the maximum score of 2.00, whereas lentogenic strains approach scores close to 0.

The values are the mean±SEM from three independent experiments.

In the ICPI test, highly virulent strains are defined as having values approaching 2.0. The ICPI values of wt BC, wt rBC, rBC-N6, and rBC-P12 were 1.6±0.02, 1.58±0.035, 1.54±0.01, and 1.52±0.045, respectively. The ICPI values of wt GBT, wt rGBT, rGBT-N6, and rGBT-P12 were 1.9±0.02, 1.88±0.035, 1.9±0.015, and 1.86±0.02, respectively (Table 1). These results indicate that the 6- and 12-nt inserts either had little effect or were slightly attenuating in the BC virus, and had little or no effect in the GBT virus. The ICPI values of rBan and rBan-ΔN6 were 1.81±0.025 and 1.68±0.135, respectively, suggesting attenuation of rBan-ΔN6 compared to its parental recombinant virus (Table 1).

The article "Effects of Naturally Occurring Six- and Twelve-Nucleotide Inserts on Newcastle Disease Virus Replication and Pathogenesis" was retracted in 2020. Reasons: manipulated images; duplicated images; concerns about the data.

### Virus replication and pathogenesis in two-week-old chickens

To study the pathogenesis of these viruses under conditions modeling natural infection, two-week-old chickens in groups of 13 were infected by the oculonasal route with 200 µL of PBS containing 10^6^ PFU of each recombinant virus per bird. Three days later, 3 birds from each group were sacrificed and virus titers in the trachea, lungs, spleen, intestine, and brain were determined (Fig. 5). Chickens infected with rBC, rBC-N6, or rBC-P12 had low virus titers in all 5 organs compared to the rGBT, rGBT-N6, and rGBT-P12 (Fig. 5). There were no consistent differences between the N6 and P12 mutants and their respective parents.

The remaining 10 chickens in each virus group were observed for clinical signs of disease until 14 days post infection (DPI). In the case of the BC virus groups, all of the chickens survived the 14-day experiment except for 1 chicken in the rBC group that died on day 10 (Fig. 6a). Chickens in the rBC group first showed mild clinical signs on 6 DPI, which increased in severity till 11 DPI and then decreased during recovery. The clinical signs included ruffled feathers, lethargy, somnolence, and self-isolation but there was no neurological signs observed. In the rBC group, chickens were severely sick, with scores substantially exceeding those of the rBC-N6 and rBC-P12 (Fig. 6b). In the rGBT, rGBT-N6, and rGBT-P12 groups, mild signs of paralysis were first observed on 3 DPI and the chickens displayed progressive neurological signs including tremors, wing drop, torticollis, opisthotonus and prostration on 4 DPI. All 10 chickens died on day 5 in rGBT, rGBT-N6, and rGBT-P12 groups (Fig. 6c, d).

In the rBan group, 1, 4, and 1 birds died on days 4, 5, and 6 DPI, respectively, and the remaining 4 birds died on 7 DPI (Fig. 6e). In the rBan-ΔN6 group, the time of death was delayed by approximately 1 day: specifically, 1, 1, 4, and 3 birds died on days 4, 5, 6, 7 DPI, respectively, and the remaining 1 bird died on 8 DPI (Fig. 6e). The disease signs include dyspnea, gasping, ruffled feathers, and self-isolation. In the clinical scoring, the scores of rBan was generally higher compared to rBan-ΔN6 except on day 6 (and 8, when all birds in each group were dead) (Fig. 6f). The mortality pattern and the clinical scores indicate a reduction in the virulence of rBan-ΔN6 compared to rBan.

The article "Effects of Naturally Occurring Six- and Twelve-Nucleotide Inserts on Newcastle Disease Virus Replication and Pathogenesis" was retracted in 2020. Reasons: manipulated images; duplicated images; concerns about the data.

## Discussion

NDV strains have natural genome lengths of 15,186 nt, 15,192 nt, and 15,198 nt. The two longer genome lengths are due to the presence of naturally-occurring 6-nt and 12-nt inserts in, respectively, the 5′ (downstream) non-translated region of the N gene and in the coding sequence for the P and V proteins. We evaluated the effects of these inserts by introducing consensus 6- and 12-nt inserts into the NDV strains BC and GBT, which are genetically closely related but differ in pathotype. Specifically, BC is a moderately virulent strain whereas GBT is a highly virulent strain used as a standard challenge virus in the U.S. We also deleted the 6-nt insert from the naturally-occurring 15,192-nt genome-length virulent NDV strain Ban, to evaluate its effect on replication and pathogenicity.

We analyzed the parental and mutant viruses for a number of features. *In vitro* growth was analyzed by multi-cycle growth kinetics and plaque size. Possible effects on N gene expression due to the presence of the N6 insert in the downstream non-translated region were evaluated by Western blot analysis of the N protein accumulation. Possible effects on P gene function due to the P12 insert, which adds four aa to P and V, were evaluated for the strain BC using a minigenome system. Virulence was scored by the standard MDT and ICPI tests with chicken eggs and one-day-old chicks, respectively. In addition, pathogenicity in two-week-old chickens was evaluated by replication, tropism, clinical disease, and mortality. Different results were obtained with the three different strains.

With the virulent strain GBT, the introduction of the 6-nt insert into the N gene, or the 12-nt insert into the P gene, had no discernible effect in any of the assays, including *in vitro* growth, N gene expression, P protein function, MDT, ICPI, and pathogenicity in two-week-old chickens. One possibility is that the very high level of virulence of the GBT strain obscured possible subtle effects of the inserts.

With the mesogenic strain BC, the introduction of these inserts did not significantly affect the growth kinetics in DF-1 cells. These results indicate that insertion of 6 nt or 12 nt into a 15,186-nt genome-length virus did not result in a growth advantage, but rather was neutral. The plaque sizes of the parental and mutant viruses were similar, suggesting that these inserts do not affect growth sufficient to result in observable difference in plaque size. No effects were observed in N gene expression or P protein function. There was no difference in MDT, but the presence of the inserts was associated with a somewhat reduced ICPI score, indicative of attenuation. Also, the inserts did not reduce BC replication in two-week-old birds but they did reduce clinical disease and mortality. Thus, the N6 and P12 inserts were associated with reduced virulence, and this effect did not appear to be due to a reduction in replication *in vivo*.

The article "Effects of Naturally Occurring Six- and Twelve-Nucleotide Inserts on Newcastle Disease Virus Replication and Pathogenesis" was retracted in 2020. Reasons: manipulated images; duplicated images; concerns about the data.

With the virulent strain Ban, deletion of the naturally-occurring 6-nt “insert” from the N gene slightly lowered replication *in vitro*, decreased virulence based on MDT, ICPI, and clinical disease and mortality in two-week-old birds, but no effect was observed in N gene expression.

Thus, while the inserts did not detectably affect strain GBT, they did affect the pathogenicity of strains BC and Ban. However, the effects were not consistent with regard to associating the presence of an insert with increased or decreased virulence. Specifically, whereas the insertion of N6 or P12 into the 15,186-nt genome of BC (to create a 15,192-nt or 15,198-nt genome, respectively) resulted in slight attenuation, the converse manipulation, namely the removal of the 6-nt “insert” from the 15,192-nt genome of strain Ban (to create a 15,186-nt genome) also resulted in attenuation. These results suggest that genome-length is a fitness controlling parameter. Any change in the naturally-occurring genomes – whether to add inserts or remove inserts – is somewhat detrimental to the virus. Thus, the naturally-occurring inserts presumably existed evolutionarily because they provide some selective advantage to that particular strain.

It was somewhat surprising that the insertion or removal of these short nt sequences would have a detectable effect on virulence, given the very small incremental change in genome-length conferred by the insertion or deletion of a 6-nt of 12-nt insert. It might have been expected that these inserts would affect expression of the respective gene or, in the case of the P12 insert that inserted 4 aa into P and V, the function of the respective proteins. Surprisingly, neither effect was observed. This is offered with the caveat that we did not directly evaluate V protein function. It appears that both proteins accommodate this aa insertion without much alteration in the phenotype of the virus. In addition, the effects were not specific to the N or P gene, and instead the effects were similar to N6 or P12. It may be that these inserts have some effect on genomic RNA folding, or on the hexamer organization of the nucleocapsid.

The article "Effects of Naturally Occurring Six- and Twelve-Nucleotide Inserts on Newcastle Disease Virus Replication and Pathogenesis" was retracted in 2020. Reasons: manipulated images; duplicated images; concerns about the data.

The origin of these inserts in nature is unknown, although they appear to have been introduced after 1960 [11], [29], it is possible that NDV strains with genome lengths of 15,192 nt and 15,198 nt existed in nature before 1960 but were not identified due to lack of extensive nucleotide sequencing. The size of each insert conforms to the “rule of six” [4], [30]. The nucleotide sequence of the inserts shows some variation among strains, indicating that the length of the insert is more important than the sequence. The likeliest mechanism of introduction of these inserts would be polymerase stuttering, with the rule of six placing a strong selective pressure for inserts to conform to the rule. There is evidence of genome-length variation in other APMVs. For example, APMV-2 strains Yucaipa and England have genome lengths of 14,904 nt, strain Kenya has a genome-length of 14,196 nt, and strain Bangor has a genome-length of 15,024 nt [31]. In APMV-3, strain Wisconsin has a genome-length of 16,182 nt compared to 16,272 nt for strain Netherlands [32]. In APMV-4, strain Delaware has a genome-length of 15,048 nt compared to 15,054 nt for strain Hong Kong [33]. In APMV-6, strain Hong Kong has a genome-length of 16,236 nt compared to 16,230 nt for strain IT4524-2 [34]. Thus, variations in genome lengths among members of genus *Avulavirus* was known, but the importance of this variation was not known.

The virus strains that naturally contain these inserts (namely, the 15,192-nt and 15,198-nt genome-length) differ substantially in nucleotide sequence from viruses that lack these inserts (the 15,186-nt genome-length) (Table S1). Strains BC and GBT (15,186-nt genome-length) share 99.1% nt sequence identity. Similarly, strains BC and GBT (both belong to genotype II of class II) share substantial identity with other 15,186-nt strains, including those of genotype I (e.g., Ulster; 90.4 and 90.7%, respectively), II (LaSota; 97.0 and 97.5%), III (Mukteswar, 87.9 and 88.1%), and IV (Herts 33, 88.0 and 88.3%). In contrast, strains BC and GBT share less identity with NDV class II strains that possess the additional 6 nt, such as: genotype V (Largo; 85.4 and 85.6%), VI (Fontana; 85.5 and 85.7%), VII (ZJ1; 83.4 and 83.6%), VIII (QH1; 84.5 and 84.6%), IX (F48E8; 87.9 and 88.1%), and XI (MG 725 08; 82.6 and 82.8%). Strains BC and GBT also share less nt identity with class I viruses, such as Alaska 415 (72.6 and 72.6%) and JS10 (72.5 and 72.5%). Thus, the 15,186-nt viruses of class II, genotypes I, II, III, and VI appear to form one relatively highly related group, with 88–99% nt identity, whereas viruses with longer genomes, of class II genotypes V, VI, VII, VIII, and IX, as well as class I, generally more divergent from strains BC and GBT, with only 72–85% identity (except for genotype IX, 88%).

The article "Effects of Naturally Occurring Six- and Twelve-Nucleotide Inserts on Newcastle Disease Virus Replication and Pathogenesis" was retracted in 2020. Reasons: manipulated images; duplicated images; concerns about the data.

The ecology and evolution of NDV is not well understood. Currently, the circulation of all three genome-length viruses (15,186-nt, 15,192-nt, and 15,198-nt) in bird populations indicate their successful establishment and survival. The NDV strains of genome-length 15,186-nt are a well-studied group that include well-defined lentogenic, mesogenic and velogenic pathotypes. Although the 15,192-nt genome-length NDV are isolated frequently from outbreaks in poultry in recent years, the spectrum of virulence within this group of viruses remains to be studied comprehensively. The viruses with genome-length 15,198-nt are lentogenic in nature and are frequently isolated from shorebirds and waterfowl [16]–[20]. However, the pigeon-origin NDV strains (pigeon paramyxoviruses) contain a genome-length of 15,192-nt and a polybasic fusion protein cleavage site sequence but are not pathogenic to chickens [35]. There are also cases in which NDV strains that phylogenetically cluster to 15,192-nt genome-length viruses, containing a polybasic fusion protein cleavage site sequence are isolated from apparently healthy chickens [36], [37]. These natural infections in birds indicate that the host species may be playing a major role in the evolution of NDV. The wider phylogenetic distance among the 15,186-nt, 15,192-nt, and 15,198-nt genome-length NDV strains points to a possibility that these genome-length viruses might have originated independently. Future studies on extensive phylogenetic analyses of NDV genomes are necessary to determine the time of divergence of different genome-length viruses in evolution.

In summary, our results showed that the 6-nt and 12-nt inserts did not detectably affect N gene expression or P protein function. The inserts had no effect on the replication or virulence of the highly virulent GBT strain. They also had no significant effect on replication of strain BC *in vivo*, but resulted in a modest degree of attenuation. We also deleted a naturally-occurring 6-nt insertion in the N gene from a highly virulent 15,192-nt genome-length virus, strain Ban. This resulted in reduced replication *in vitro* and reduced virulence *in vivo*. Thus, although these inserts had no evident effect on gene expression, protein function, or replication *in vivo*, they did affect virulence in two of the three tested strains. These results suggest that NDV has evolved to produce different genome lengths which is optimal for the replication and pathogenesis of that strain in a particular host and environment.

The article "Effects of Naturally Occurring Six- and Twelve-Nucleotide Inserts on Newcastle Disease Virus Replication and Pathogenesis" was retracted in 2020. Reasons: manipulated images; duplicated images; concerns about the data.

## Supporting Information

Table S1 Per cent nucleotide sequence identities among the genome sequences of representative Newcastle disease virus strains.
(DOCX)
